The article "Hyal1 Expression in Colorectal Carcinoma Cell Migration and Invasiveness: Significance and Mechanism" was retracted in 2023. Reasons: signs of a paper mill; suspected computer-generated content; unreliable results or conclusions; concerns about the data.

# Hyal1 Expression in Colorectal Carcinoma Cell Migration and Invasiveness: Significance and Mechanism

**DOI:** 10.1155/2022/4418300

**Published:** 2022-07-05

**Authors:** Shuangshuang Zhao, Junhui Zhao, Ni Zhang

**Affiliations:** ^1^Department of Radiation Oncology, Hangzhou Cancer Hospital, Hangzhou, Zhejiang 310002, China; ^2^College of Basic Medicine, Zhejiang Chinese Medical University, Hangzhou, Zhejiang 310002, China

## Abstract

**Objective:**

To clarify the significance of hyaluronidsase 1 (Hyal1) expression in colorectal carcinoma (CRC) and its impact on tumor cell migration and invasiveness.

**Methods:**

Human CRC cell lines SW480, HCT116, and SW620 were purchased, ELISA and western blot were used to detect the expression of Hyal1 in cells, CCK-8 assay to detect cell proliferation ability, cell scratch assay to check cell migration rate, and cell invasion was detected by the transwell assay. The correlation of Hyal1 with CRC cell migration and invasiveness capacities was analyzed.

**Result:**

ELISA results showed that supernatant Hyal1 level was the lowest in SW480, highest in HCT116, with the level in SW620 in between (*P* < 0.05). No evident difference was identified by western blot in Hyal1 protein expression among the three cells (*P* > 0.05). The cell scratch assay and transwell assay showed that the migration and invasion ability of HCT116 cells was higher than that of SW620 (*P* < 0.05). In vitro, Hyal1 had a synergistic relationship with the invasiveness and migration capacities of CRC cells (*P* < 0.05).

**Conclusion:**

Hyal1 is elevated in CRC and is consistent with the invasiveness and metastasis abilities of CRC cells. It is hoped that this research can provide reference for future prevention and treatment of CRC.

## 1. Introduction

Colorectal carcinoma (CRC) is one of the most common malignant neoplastic diseases, second only to lung and gastric carcinomas. Statistics show that in 2018, there were over 1.8 million new CRC cases around the world, with the majority of them aged over 40 [1]. Recent years have witnessed the growing incidence of CRC, and it is expected that by 2030, CRC will become the malignancy with the highest incidence [2]. At present, the pathogenesis of CRC has not yet been fully clarified, but it is believed to be strongly linked to environment, diet, genetics, and other factors in clinical practice [3]. The disease usually has strong concealment in the early stage of illness, which may only be manifested as diarrhea, constipation, and other changes in defecation habits, and as the disease progresses, bloody stools and fatigue begin to appear [4]. This also directly leads to the fact that most CRC patients have reached the middle and late stage at the time of diagnosis when CRC has a high possibility of metastasis and invasiveness, which seriously increases the difficulty of treatment and leads to a bleak prognosis of patients [5]. According to the survey, the 5-year mortality rate of advanced CRC patients is as high as 60–80%, with approximately 900,000 deaths each year due to CRC [6]. Due to the high morbidity and mortality of the disease, clinical work in recent years has been focused on finding new diagnostic and treatment options for CRC, with a focus on molecular pathogenesis.

The article "Hyal1 Expression in Colorectal Carcinoma Cell Migration and Invasiveness: Significance and Mechanism" was retracted in 2023. Reasons: signs of a paper mill; suspected computer-generated content; unreliable results or conclusions; concerns about the data.

In 2016, a phase IB clinical study on PEGylation of recombinant human hyaluronidase PH20 (PEGPH20) in the treatment of pancreatic carcinoma found that via removing hyaluronic acid from the extracellular matrix, PEGPH20 can dilate pancreatic carcinoma blood vessels, and increase the gap between tumor vascular endothelial cells and fenestrations to achieve chemosensitization effects [7], which has aroused people's attention to hyaluronidases (Hyals) in neoplastic diseases. Hyaluronidase 1 (Hyal1), a vital member of the five Hyals, has been shown to promote cell proliferation and motility by accelerating vesicle motility [8], but its relationship with CRC is still unclear. In previous studies, we found that Hyal1 is the only Hyals that can be detected in plasma, and its expression level is closely related to the disease changes of CRC [9]. A large number of basic studies and clinical trials have shown that the expression level of Hyal1 is positively correlated with the occurrence and development of CRC. Bouga et al. found that Hyal1, Hyal2, Hyal3, and PH20 were obviously overexpressed in CRC and normal tissue extracts, with the highest expression in the late stage [10]. From the clinical data, it can be seen that Hyal1 promotes CRC occurrence and development. However, there is no other related research that can further confirm the influencing mechanism of Hyal1 on CRC. Therefore, we initially analyze the role of Hyal1 in CRC in the face of the increasing incidence of CRC by detecting Hyal1 in colon carcinoma (CC) cell lines with different metastatic potential.

## 2. Data and Methods

### 2.1. Cell Data

SW480, SW620, and HCT116, which were human CRC cell strains, were supplied by the Cell Bank of Chinese Academy of Sciences Shanghai Branch. The above cells were then cultured. The medium was RPM1640 plus fetal bovine serum diluted at 10% as well as penicillin-streptomycin at the concentration of 100 U/ml, and the conditions were 37°C and 5% CO_2_ in air.

### 2.2. Detection of Hyal1 Levels in Cells

ELISA and western blot detected supernate Hyal1 expression. ELISA kits were provided by Wuhan Fine Biotech, and the operation process was carried out in strict accordance with the manufacturer's recommendations. In addition, RIPA lysate was used to lysate the cells and extract the total protein. After the purity was verified, the proteins were transferred to PVDF membranes via SDS-PAGE electrophoresis, and the primary antibodies Hyal1 (1 : 500) and *β*-actin (1 : 1,000) were added and blocked overnight at 4°C. After the primary antibody incubation overnight, the membrane was washed with TBST five times for a total of 35 min. The second antibody (1 : 1,000) was added for 1 hour incubation. Then, the secondary antibody is also washed with TBST five times and the gray value of proteins was analyzed by ImageJ software.

The article "Hyal1 Expression in Colorectal Carcinoma Cell Migration and Invasiveness: Significance and Mechanism" was retracted in 2023. Reasons: signs of a paper mill; suspected computer-generated content; unreliable results or conclusions; concerns about the data.

### 2.3. Cell Multiplication Testing

Cells (5 × 10^3^/well) were inoculated in the wells of a 96-well plate for 6 days of cultivation, and the solution was changed every 2 days. Ten microliters of CCK-8 reagent were added to each well at an interval of 24 h and incubated for 2 h at 37°. The absorbance_450nm_ value was read with the use of a microplate reader, and the growth curve was plotted.

### 2.4. Cell Migration Testing

After the cells were digested and plated, 5 × 10^5^ cells were added to each well. When the cells covered the bottom of the plate, the 20 *μ*L pipette tip was used to draw lines vertically. After the old medium was aspirated, PBS was applied twice to remove the cells scratched by the pipette tip. Then, a culture medium comprising 1% FBS was added to each well, and the cell migration distance was observed and the mobility was calculated after 24 hours of continuous culture.

### 2.5. Cell Invasiveness Testing

The logarithmic growth cells were digested, resuspended, and inoculated into the upper chamber of the transwell chamber at 2.5 × 10^5^/ml. A complete culture medium (500 *μ*L) was added to the lower chamber for 48 h. The chamber was removed, Matrigel was wiped with *Q*-tips, and the transmembrane cells were stained with 95% ethanol and 1% crystal violet after washing with PBS, for microscopical counting.

### 2.6. Statistical Processing

Data was processed by SPSS22.0. Quantitative data were recorded by (*χ* ± *s*), and the differences were determined via independent sample *t*-test. The comparison of three and more groups used one-way ANOVA. *P* < 0.05 was the threshold of significance.

## 3. Results

### 3.1. Hyal1 Expression in CRC Cells

ELISA showed no distinct difference in supernatant Hyal1 expression in HCT116 and SW620 cells at 48 h (*P* > 0.05), higher than SW480 (*P* < 0.05). At 72 h, supernatant Hyal1 level was the lowest in SW480, highest in HCT116, with the level in SW620 in between (*P* < 0.05). No evident difference was identified by western blot in Hyal1 protein expression among the three cells (*P* > 0.05) (Figure 1).

The article "Hyal1 Expression in Colorectal Carcinoma Cell Migration and Invasiveness: Significance and Mechanism" was retracted in 2023. Reasons: signs of a paper mill; suspected computer-generated content; unreliable results or conclusions; concerns about the data.

### 3.2. Impacts of Hyal1 on CRC Cell Proliferation

As indicated by CCK-8 experimental results, the three cells had similar proliferation ability (*P* > 0.05) (Figure 2).

### 3.3. Impacts of Hyal1 on CRC Cell Migration

In the scratch assay, highest cell migration was observed in HCT116 and lowest in SW480, with that of SW620 in between (*P* < 0.05) (Figure 3).

### 3.4. Impacts of Hyal1 on CRC Cell Invasion

Similarly, the Transwell test showed highest invasiveness in HCT116, followed by SW620, with that of SW480 being the lowest (*P* < 0.05) (Figure 4).

## 4. Discussion

As one of the most frequently occurring tumors in clinical practice, the potential threat of CRC to patients deserves clinical attention [11, 12]. At present, the research on small molecule RNAs in neoplastic diseases is the focus of clinical research. As an important substance participating in multiple life cycles of human organs, tissues and cells, the significance of small molecule RNA research lies in the following aspects: (1) they are expected to become new clinical markers that can assist in assessing the occurrence and development of tumour diseases; (2) as molecular therapeutic targets for neoplastic diseases, they can be used to optimize the killing effect of current radiotherapy and chemotherapy on tumor cells [13, 14]. For Hyal1, it has been confirmed to present abnormal expression in bladder carcinoma, pancreatic carcinoma and other diseases [15–17], but there is still a lack of relevant studies to confirm its exact role in occurrence and development of CRC. Therefore, this study, by exploring the connection between Hyal1 and CRC, has great reference significance for clinical practice, which can also lay a foundation for follow-up research.

In this experiment, we found that Hyal1 expression had a synergistic effect with the invasiveness and migration of CRC cells, and the cells with higher Hyal1 expression had significantly stronger activity, which shows that highly expressed Hyal1 plays the role of oncogene in CRC. However, Hyal1 was found to be in a low expression state in the studies of Puissant et al. [18, 19], contrary to our findings. Based on previous studies, we believe that whether Hyal1 promotes or inhibits tumor formation depends on two factors, one is the tumor type, and the other is the concentration of Hyal1. Lokeshwar et al. showed that Hyal1 inhibited or promoted the formation of prostate carcinoma (PC) depending on the level of Hyal1 in PC tissues and cells. At the background level, Hyal1 promotes the growth, invasiveness, and vascular formation of PC, but when Hyal1 is overexpressed by gene transfection (Hyal1 > 100 milliunits/10^6^ cells), it inhibits PC formation and growth via inducing apoptosis [20]. When Jacobson tested Hyal1 expression in a Hyal1-overexpressed model of rabbit CC cells, it was found that Hyal1 reached 220–360 milliunits/10^6^ cells, far exceeding the background level of 20 milliunits/10^6^ cells of CC cells [21]. Therefore, in this study, the high level of Hyal1 is consistent with the high invasiveness and metastasis capacities of CC, which preliminarily indicates that upregulated Hyal1 promotes the occurrence and development of CRC.

The article "Hyal1 Expression in Colorectal Carcinoma Cell Migration and Invasiveness: Significance and Mechanism" was retracted in 2023. Reasons: signs of a paper mill; suspected computer-generated content; unreliable results or conclusions; concerns about the data.

Inhibition of Hyal1 has been shown to inhibit tumor formation of PC and bladder carcinoma, where Hyal1 overexpression is most typical [22]. Sulfated hyaluronan (sHA), as an inhibitor of Hyal1, can inhibit PC cell growth, migration, and infiltration, downregulate Bcl-2 and p-Bad to induce apoptosis, and downregulate androgen receptor activation, NFkb activation, and VEGF expression via inhibiting the PI3K-AKT axis, which has been verified in animal models [23]. In bladder carcinoma, sHA also inhibits tumor formation by suppressing PI3K-AKT axis [24]. Therefore, the inhibition of Hyal1 is a novel approach for the treatment of Hyal1-overexpressed tumors, and inhibiting Hyal1 provides a new idea and method to treat CRC. However, at present, sHA is the only one known to inhibit cell function among Hyal1 inhibitors [25]. In the future, we plan to apply the Hyal1 inhibitor sHA to CC cells and detect its inhibition on CRC cell function. Besides, we need more experiments to verify Hyal1 expression in CRC, and further confirm its impacts on CRC *in vivo* through tumorigenesis experiments in nude mice.

## 5. Conclusion

This study finds that Hyal1 expression remains at a high level in CRC, which is consistent with the capacities of CRC cells to invade and metastasize. Also, it was initially shown that upregulated Hyal1 promoted the occurrence and development of CRC. Inhibition of Hyal1 inhibits tumor formation of CRC. It is hoped that this research can provide reference for future prevention and treatment of CRC.

## Figures and Tables

**Figure 1:** Hyal1 expression in CRC cells. (a) The expression of Hyal1 was detected by ELISA. (b) The expression of Hyal1 was detected by western blot. Compared with SW480, ^*∗*^*P* < 0.05. Compared with SW620, ^#^*P* < 0.05.

**Figure 2:** Impacts of Hyal1 on CRC cell proliferation.

**Figure 3:** Impacts of Hyal1 on CRC cell migration. (a) Cell scratch assay. (b) Cell migration rate. Compared with SW480, ^*∗*^*P* < 0.05. Compared with SW620, ^#^*P* < 0.05.

**Figure 4:** Impacts of Hyal1 on CRC cell invasion. (a) Invasive cell staining. (b) Number of cells invaded. Compared with SW480, ^*∗*^*P* < 0.05. Compared with SW620, ^#^*P* < 0.05.

The article "Hyal1 Expression in Colorectal Carcinoma Cell Migration and Invasiveness: Significance and Mechanism" was retracted in 2023. Reasons: signs of a paper mill; suspected computer-generated content; unreliable results or conclusions; concerns about the data.

## Data Availability

The data can be obtained from the author upon reasonable request.
